The article "Mathematical Analysis of Two Waves of COVID-19 Disease with Impact of Vaccination as Optimal Control" was published in 2022. Journal: Comput Math Methods Med.

# Mathematical Analysis of Two Waves of COVID-19 Disease with Impact of Vaccination as Optimal Control

**DOI:** 10.1155/2022/2684055

**Published:** 2022-04-14

**Authors:** P. K. Santra, D. Ghosh, G. S. Mahapatra, Ebenezer Bonyah

**Affiliations:** ^1^Maulana Abul Kalam Azad, University of Technology, Kolkata 700064, India; ^2^Department of Mathematics, National Institute of Technology, Karaikal 609609, Puducherry, India; ^3^Department of Mathematics Education, Aken Appiah Menka University of Skills Training and Entrepreneurial Development, Kumasi 233243357651, Ghana

## Abstract

This paper is devoted to answering some questions using a mathematical model by analyzing India's first and second phases of the COVID-19 pandemic. A new mathematical model is introduced with a nonmonotonic incidence rate to incorporate the psychological effect of COVID-19 in society. The paper also discusses the local stability and global stability of an endemic equilibrium and a disease-free equilibrium. The basic reproduction number is evaluated using the proposed COVID-19 model for disease spread in India based on the actual data sets. The study of nonperiodic solutions at a positive equilibrium point is also analyzed. The model is rigorously studied using MATLAB to alert the decision-making bodies to hinder the emergence of any other pandemic outbreaks or the arrival of subsequent pandemic waves. This paper shows the excellent prediction of the first wave and very commanding for the second wave. The exciting results of the paper are as follows: (i) psychological effect on the human population has an impact on propagation; (ii) lockdown is a suitable technique mathematically to control the COVID spread; (iii) different variants produce different waves; (iv) the peak value always crosses its past value.

## 1. Introduction

The novel coronavirus (COVID-19) has spread in almost all parts of the world at the pandemic level. Many researchers [1, 2] have developed different models incorporating the hazards of COVID-19 pandemic. Atangana and Araz [3] describe the model and forecast the spread of COVID-19 in Africa and Europe. Wu et al. [4] form a COVID-19 model on the use of social distancing personal protection in Ontario, Canada. Aldila et al. [5] used the community awareness as a control scheme to minimize the transmission of COVID-19 outbreak. Sen and Ibeas [6] used vaccination [7] and antiviral to control the pandemic of COVID-19. Some researchers [8, 9, 30, 32, 33, 36, 39] have discussed the effect of COVID-19 in society and optimal policy in different countries.

After the initial outbreak, COVID-19 continued to spread to all provinces in India. India has controlled [10] the rate of spread of COVID-19 after the first phase of the outbreak. However, due to the negligence of people, it spread quickly more than the first variant in the second wave [11, 12]. Mathematical modelling is used to predict the number of active cases, disease spread, and duration of this pandemic and estimate the impact of measures during disease outbreaks. Ghosh et al. [13] described the transmission of COVID-19 outbreak in India based on the 1st wave. The second wave of the pandemic has come at the end of January 2021 in different countries including India; in this respect, Ershkov and Rachinskaya [14] and Glass [15] both perform a model to describe the second wave of COVID-19.

This article presents a mathematical model that describes the evolution of the COVID-19 in India using the actual data in two phases, 1^st^ phase from March 23 to December 31, 2020, and 2^nd^ phase of daily update confirmed cases, recovered, and deaths in India, in order to estimate the parameters of the model and then predict the severity of the possible infection in the coming months. Using this method, we can estimate the size of the population at risk in India and justify the growing number of new confirmed cases. With the aim to reduce the population at risk in India, we investigate an optimal control strategy by adopting vaccine which makes it very optimal, and this study may be more practical to use in developing countries. In this study, we are trying to answer some questions. How many waves come? What will be the peak value of the consequence wave? What is the effect of lockdown on COVID control? Is there any effect of fear in propagation? We are given some answers to these questions using a mathematical model.

The contents of this study are organised as follows. The first section has laid the context of the work. The second section discusses the preparation of the model and its basic properties.  Section 3 finds the equilibrium points and checks the stability like local and global. The fourth section discusses the nonexistence of a periodic solution. The fifth section forms a COVID-19 model with the concept of optimal control. The sixth section presents the results for different waves in respect to India. Finally, section seven concludes this study and presents the precaution and future directions for this research work.

## 2. Novel Coronavirus Model with Basic Properties

Already in the literature, there are some papers to understand the dynamics of novel coronavirus spread [13, 16–18, 31, 34, 35, 37, 38, 40, 41]. This coronavirus model proposes to fill the inadequacy of previous studies for analyzing the spread dynamics incorporating the effect on human consciousness of the novel COVID-19. Based on the medical practitioners' instructions, regular hand wash, nose and mouth cover, safe distancing, etc. affect the transmission rate. We consider *α* as a representative of hand wash, nasal and oral cover, and social distancing in the proposed coronavirus model, and hence, increasing disease transmission means that such instructions are not followed properly. This model also considers the consciousness of the disease as a parameter, i.e., the parameter *δ* measures the psychological or inhibitory effect. Furthermore, this model considers a saturated incidence rate *g*(*I*_*u*_)*S* for COVID-19 pandemic model, when *I*_*u*_ gets larger, i.e., *g*(*I*_*u*_) = *αI*_*u*_/(1 + *δI*_*u*_) tends to be overloaded, where infection force of the disease is calculated by *αI*_*u*_, and 1/(1 + *δI*_*u*_) measures the reticence effect from the observable change of the susceptible individuals when their number increases or from the crammed effect of the infected individuals. For COVID-19, the proposed rate of incidence [19–21] seems more justifiable compared to the other incidence rate, because it includes the detectable change and cramming effect of the infected individuals and prevents the unboundedness of the association rate by choosing apt and relevant parameters.

At time *t*, let *S*(*t*), *I*_*u*_(*t*), *I*_*k*_(*t*), and *R*(*t*) be the densities of susceptible population (*S*), unrevealed infected population (*I*_*u*_) which spread the disease, known infected population (*I*_*k*_) in isolated ward for treatment not spreading the disease, and recover population (*R*), respectively. Our important conjecture for this model is that the disease spread by unrevealed infected populations and COVID has a psychological effect on the human population.

The mathematical form of the novel coronavirus transmission as discussed above takes the following form:

(1) $$\begin{array}{c} \begin{array}{c} \frac{dS}{dt}=\Lambda -\frac{\alpha SI_{u}}{1+\delta I_{u}}-d_{1}S,\\ \frac{dI_{u}}{dt}=\frac{\alpha SI_{u}}{1+\delta I_{u}}-\beta I_{u}-d_{1}I_{u},\\ \frac{dI_{k}}{dt}=\beta I_{u}-\gamma I_{k}-d_{2}I_{k},\\ \frac{dR}{dt}=\gamma I_{k}-d_{1}R. \end{array} \end{array}$$

Here, *N*(*t*) = *S*(*t*) + *I*_*u*_(*t*) + *I*_*k*_(*t*) + *R*(*t*) stands for the total number of human community in the system at time *t*. The proposed COVID-19 pandemic model will analyse with the following initial densities:

(2) $$\begin{array}{c} S\left(0\right)=S_{0},R\left(0\right)=R_{0}>0,\\ \;I_{u}\left(0\right)=I_{u_{0}},I_{k}\left(0\right)=I_{k_{0}}\geq 0. \end{array}$$

The flow diagram of the proposed COVID-19 pandemic model is presented in Figure 1. The model parameters with their assumed and estimated values from the real data of India during the time span of 1st February to 6th June 2021 are described in Table 1.

Since in this novel coronavirus model the variable *R*(*t*) has no effect in dynamics of the system, we eliminate the last equation from the pandemic model (1) for the dynamical analysis. Hence, the dynamical study of COVID-19 system is considered from India's perspective using the following mathematical model:

(3) $$\begin{array}{c} \frac{dS}{dt}=\Lambda -\frac{\alpha SI_{u}}{1+\delta I_{u}}-d_{1}S, \end{array}$$

(4) $$\begin{array}{c} \frac{dI_{u}}{dt}=\frac{\alpha SI_{u}}{1+\delta I_{u}}-\beta I_{u}-d_{1}I_{u}, \end{array}$$

(5) $$\begin{array}{c} \frac{dI_{k}}{dt}=\beta I_{u}-\gamma I_{k}-d_{2}I_{k}. \end{array}$$

### 2.1. Nonnegativity of Solution of COVID-19 Model

**Theorem 1 .**

Every solution of COVID-19 system (1) with initial conditions (2) exists in the interval [0, ∞) and *S*(*t*) > 0, *I*_*u*_(*t*) ≥ 0, *I*_*k*_(*t*) ≥ 0, and *R*(*t*) > 0 for all *t* ≥ 0.

**Proof**

Since the right hand side of COVID-19 model (1) is continuous and locally Lipschitzian, then the solution (*S*(*t*), *I*_*u*_(*t*), *I*_*k*_(*t*), *R*(*t*)) of (1) with respect to the initial conditions is unique on [0, *ξ*), where 0 < *ξ* < +∞.

From the model (1) and using the initial conditions, we have

(6) $$\begin{array}{c} \frac{dS}{dt}=\Lambda -\left(d_{1}+\frac{\alpha I_{u}\left(t\right)}{1+\delta I_{u}\left(t\right)}\right)S\left(t\right). \end{array}$$

We thus have

(7) $$\begin{array}{c} \frac{d}{dt}\left[S\left(t\right)\exp\left\{d_{1}t+\int_{0}^{t}\frac{\alpha I_{u}\left(s\right)}{1+\delta I_{u}\left(s\right)}ds\right\}\right]=\Lambda \exp\left\{d_{1}t+\int_{0}^{t}\frac{\alpha I_{u}\left(s\right)}{1+\delta I_{u}\left(s\right)}ds\right\}. \end{array}$$

Hence,

(8) $$\begin{array}{c} S\left(t\right)\exp\left\{d_{1}t+\int_{0}^{t}\frac{\alpha I_{u}\left(s\right)}{1+\delta I_{u}\left(s\right)}ds\right\}-S\left(0\right)=\int_{0}^{t}\Lambda \exp\left\{d_{1}t+\int_{0}^{t}\frac{\alpha I_{u}\left(\omega \right)}{1+\delta I_{u}\left(\omega \right)}d\omega \right\}dt, \end{array}$$

so that

(9) $$\begin{array}{c} S\left(t\right)=S_{0}\exp\left[-\left\{d_{1}t+\int_{0}^{t}\frac{\alpha I_{u}\left(s\right)}{1+\delta I_{u}\left(s\right)}ds\right\}\right]+\exp\left[-\left\{d_{1}t+\int_{0}^{t}\frac{\alpha I_{u}\left(s\right)}{1+\delta I_{u}\left(s\right)}ds\right\}\right]\times \left[\int_{0}^{t}\Lambda \exp\left\{d_{1}t+\int_{0}^{t}\frac{\alpha I_{u}\left(\omega \right)}{1+\delta I_{u}\left(\omega \right)}d\omega \right\}dt\right]>0. \end{array}$$

The second equation of the model (1) yields *dI*_*u*_/*dt* ≥ −(*β* + *d*_1_)*I*_*u*_(*t*) which gives *I*_*u*_(*t*) ≥ *I*_*u*_0__exp[−(*β* + *d*_1_)*t*] ≥ 0.

From the third equation of system (1), we get *dI*_*k*_/*dt* ≥ −(*γ* + *d*_2_)*I*_*k*_ which gives *I*_*k*_(*t*) ≥ *I*_*k*_0__exp[−(*γ* + *d*_2_)*t*] ≥ 0.

The last equation of the system (1) yields *dR*/*dt* ≥ −*d*_1_*R*(*t*) which gives *R*(*t*) ≥ *R*_0_exp[−(*d*_1_)*t*] > 0.

Therefore, we can see that *S*(*t*), *R*(*t*) > 0, and *I*_*u*_(*t*), *I*_*k*_(*t*) ≥ 0, ∀*t* ≥ 0.

This completes the proof.

### 2.2. Invariant Region of Solutions of COVID-19 Model

**Theorem 2 .**

All solutions of COVID-19 system (1) in ℝ_+_^4^ are bounded and lie in the region *Ω* defined by *Ω* = {(*S*, *I*_*u*_, *I*_*k*_, *R*) ∈ ℝ_+_^4^ : 0 < *N*(*t*) ≤ *Λ*/*μ*} as *t*⟶∞, where *μ* = min{*d*_1_, *d*_2_}.

**Proof**

Assume (*S*(*t*), *I*_*u*_(*t*), *I*_*k*_(*t*), *R*(*t*)) be any solution of system (1). Now, we consider a function like *N*(*t*) = *S*(*t*) + *I*_*u*_(*t*) + *I*_*k*_(*t*) + *R*(*t*). Differentiating both sides with respect to *t*, we have

(10) $$\begin{array}{c} \frac{dN\left(t\right)}{dt}=\frac{dS\left(t\right)}{dt}+\frac{dI_{u}\left(t\right)}{dt}+\frac{dI_{k}\left(t\right)}{dt}+\frac{dR\left(t\right)}{dt},\\ \frac{dN\left(t\right)}{dt}=\Lambda -d_{1}S-d_{1}I_{u}-d_{2}I_{k}-d_{1}R,\\ \frac{dN\left(t\right)}{dt}+\mu N\left(t\right)=\Lambda -\left(d_{1}-\mu \right)S-\left(d_{1}-\mu \right)I_{u}-\left(d_{2}-\mu \right)I_{k}-\left(d_{1}-\mu \right)R. \end{array}$$

(*dN*(*t*)/*dt*) + *μN*(*t*) ≤ *Λ*, assuming *μ* = min{*d*_1_, *d*_2_}.

Then, by comparison theorem, we obtain 0 < *N*(*t*) ≤ *N*(0)*e*^−*μt*^ + (*Λ*/*μ*) and for *t*⟶∞, 0 < *N*(*t*) ≤ *Λ*/*μ*. Therefore, all solutions of coronavirus system (1) enter into the region *Ω* = {(*S*, *I*_*u*_, *I*_*k*_, *R*) ∈ ℝ_+_^4^ : 0 < *N*(*t*) ≤ *Λ*/*μ*}.

### 2.3. The Basic Reproduction Number

**Definition 1 (basic reproduction number (BRN)).**

“The BRN is defined as the number of newly infected individuals produced by a single infected individual during his or her effective infectious period when it is introduced into the susceptible population.”

Here, the BRN (*ℜ*_0_) for the proposed COVID-19 model (1) is given by

(11) $$\begin{array}{c} R_{0}=\frac{\alpha \Lambda }{\left(\beta +d_{1}\right)d_{1}}. \end{array}$$

Impact of transmission coefficient *α* from *S* to *I*_*u*_ is measured qualitatively on the coronavirus disease transmission dynamics.

Since *∂ℜ*_0_/*∂α* = *Λ*/((*β* + *d*_1_)*d*_1_) > 0, it is obvious that if *α* decreases, then BRN *ℜ*_0_ also decreases and therefore reduces the disease burden. On the other side, if *α* increase, then *ℜ*_0_ would rise leading to the rise of the infection burden, and therefore, the scenario changes to be a very harmful one.

From Figure 2, we observe that if the values of *α* increases then the value of *ℜ*_0_ also increases (both cases first wave and second wave), and after certain value of *α*, *ℜ*_0_ becomes greater than 1. From these two figures, we also observed that the second wave in India is more dangerous than the 1st wave. Our study finds that the mathematical model of this type does not predict the wave. So different waves come due to different strains of the COVID-19 virus.

## 3. Existence of Equilibrium Points and Stability

The equilibrium points of the proposed COVID-19 system (3) are (i) disease-free equilibrium point *E*_1_(*Λ*/*d*_1_, 0, 0) and (ii) endemic equilibrium *E*^∗^(*S*^∗^, *I*_*u*_^∗^, *I*_*k*_^∗^), where *S*^∗^ = ((1 + *δI*_*u*_^∗^)(*β* + *d*_1_))/*α*, *I*_*u*_^∗^ = (*αΛ* − *d*_1_(*β* + *d*_1_))/((*β* + *d*_1_)(*δd*_1_ + *α*)), and *I*_*k*_^∗^ = (*β*/(*γ* + *d*_2_))*I*_*u*_^∗^. The endemic equilibrium point exists when *ℜ*_0_ > 1.

### 3.1. Local Stability Analysis

The local stability analysis of the coronavirus model (3) is presented at the equilibrium points.

#### 3.1.1. Disease-Free Equilibrium

**Theorem 3 .**

Disease-free equilibrium point *E*_1_(*Λ*/*d*_1_, 0, 0) is locally asymptotically stable if *ℜ*_0_ < 1, marginally stable if *ℜ*_0_ = 1, and unstable if *ℜ*_0_ > 1.

The proof of this theorem is in the Appendix.

#### 3.1.2. Endemic Equilibrium

**Theorem 4 .**

Endemic equilibrium point *E*^∗^(*S*^∗^, *I*_*u*_^∗^, *I*_*k*_^∗^) is locally asymptotically stability if *ℜ*_0_ > 1.

The proof of this theorem is in the Appendix.

Therefore, up to a certain value of *α* disease-free equilibrium point is stable (Theorem 4) and beyond that value of *α* endemic equilibrium point is stable (Theorem 5).

### 3.2. Global Stability Analysis

The global stability analysis of the proposed COVID-19 model (3) is presented here.

#### 3.2.1. Disease-Free Equilibrium

**Theorem 5 .**

If *ℜ*_0_ < 1, the disease-free equilibrium *E*_1_ is globally asymptotically stable.

The proof of this theorem is in the Appendix.

#### 3.2.2. Global Stability of Endemic Equilibrium: Geometric Approach

The global stability of the endemic equilibrium *E*^∗^ will be discussed when *ℜ*_0_ > 1 using the geometric approach for global dynamics [22]. For some preliminary discussion on the geometric approach, consider the autonomous dynamical system:

(12) $$\begin{array}{c} \overset{.}{x}=f\left(x\right), \end{array}$$

where *f* : *D*⟶ℝ^*n*^, *D* ∈ ℝ^*n*^ open set and simply connected and *f* ∈ *C*^1^(*D*).

Let *A*(*x*) be an $\left(\begin{array}{c} n\\ 2 \end{array}\right)\times \left(\begin{array}{c} n\\ 2 \end{array}\right)$ matrix value function that is *C*^1^ on *D* and consider *Q* = *A*_*f*_*A*^−1^ + *AJ*^[2]^*A*^−1^, where the matrix *A*_*f*_ is (*q*_*ij*_(*x*))_*f*_ = (*∂q*_*ij*_(*x*)/*∂x*)^*T*^. *f*(*x*) = ∇*q*_*ij*_.*f*(*x*), and here, *J*^[2]^ represents the second additive compound matrix of *J*(*x*) = *D*(*x*). Let the Lozinskii measure [23] *μ* of *Q* concerning a vector norm |.| in ${\mathbb{R}}^{\left(\begin{array}{c} n\\ 2 \end{array}\right)}$ be $\mu \left(Q\right)=\underset{h⟶0^{+}}{\lim}\left(\left|I+hQ\right|-1\right)/h.$ Define a quantity ${\overset{¯}{q}}_{2}$ as ${\overset{¯}{q}}_{2}=\lim\underset{t⟶\infty }{\sup}\underset{x_{0}⟶K}{\sup}\left(1/t\right)\int_{0}^{t}\mu \left(Q\left(x\left(s,x_{0}\right)\right)\right)ds.$ We will apply the following theorem.

**Theorem 6 .**

Let *D* be simply connected, and [23] (H1) “there exists a compact absorbing set *K* ⊂ *D*,” (H2) “the system (12) has a unique equilibrium $\tilde{x}$ in *D*,” then $\tilde{x}$ of (12) is globally asymptotically stable in *D* if ${\overset{¯}{q}}_{2}<0$.

**Theorem 7 .**

The COVID-19 model (3) admits an unique endemic equilibrium which globally asymptotically stable if *ℜ*_0_ > 1.

The proof is in the Appendix.

Since disease-free equilibrium point *E*_1_(*Λ*/*d*_1_, 0, 0) is globally stable for *ℜ*_0_ < 1 and an unique endemic equilibrium point *E*^∗^(*S*^∗^, *I*_*u*_^∗^, *I*_*k*_^∗^) is globally stable for *ℜ*_0_ > 1, so there exists no limit cycle for this model. Therefore, we include Nonexistence Periodic Solution part for only the mathematical purpose for the proof in a different way.

## 4. Nonexistence Periodic Solution

This section presents suitable conditions for the COVID system (3) for nonperiodic solutions around the positive equilibria *E*^∗^ based on the criterion of [23]; let an autonomous ordinary differential equation as follows:

(13) $$\begin{array}{c} \frac{dx}{dt}=f\left(x\right), \end{array}$$

where *f* is a function in *C*^1^ in open subset of ℝ^*N*^. Let *J* = *df*/*dx* be the Jacobian matrix of system (13), and *J*^[2]^ be the matrix of $\left(\begin{array}{c} N\\ 2 \end{array}\right)\times \left(\begin{array}{c} N\\ 2 \end{array}\right)$ which represents as the second additive compound matrix [23] associated with the Jacobian matrix *J*. Let the matrix *J* = (*a*_*ij*_)_*n*×*n*_ for $i=1,2,3,\cdots \left(\begin{array}{c} N\\ 2 \end{array}\right)$, let (*i*) = (*i*_1_, *i*_2_) be the *i*th member in the lexicographic ordering of integer pairs (*i*_1_, *i*_2_) for 1 ≤ *i*_1_ ≤ *i*_2_ ≤ *n*. Then, the (*i* × *j*)^th^ element of *J*^[2]^ is

(14) $$\begin{array}{c} \left\{\begin{array}{cc} a_{i_{1}i_{1}}+a_{i_{2}i_{2}}, & \text{if }\left(i\right)=\left(j\right),\\ {\left(-1\right)}^{r+s}a_{i_{r}j_{s}}, & \text{if exactly one entry }i_{r}\text{ of }\left(i\right)\text{ does not occur in }\left(j\right)\text{ and }j_{s}\text{ does not occur in }\left(j\right)\\ 0, & \text{if neither entry from }\left(i\right)\text{ occurs in }\left(j\right). \end{array}\right. \end{array}$$

For a general 3 × 3 matrix

(15) $$\begin{array}{c} J=\left(\begin{array}{ccc} a_{11} & a_{12} & a_{13}\\ a_{21} & a_{22} & a_{23}\\ a_{31} & a_{32} & a_{33} \end{array}\right), \end{array}$$

its second additive compound matrix *J*^[2]^ is

(16) $$\begin{array}{c} J^{\left[2\right]}=\left(\begin{array}{ccc} a_{11}+a_{22} & a_{23} & -a_{13}\\ a_{32} & a_{11}+a_{33} & a_{12}\\ -a_{31} & a_{21} & a_{22}+a_{33} \end{array}\right). \end{array}$$

In this case, (1) = (1, 2), (2) = (1, 3), (3) = (2, 3).

**Theorem 8 .**

Bendixson's criterion [23]: a simple closed rectifiable function cannot exist which is invariant under the system (13) for *x* ∈ ℝ^*n*^ if any one of the following conditions is satisfied:

- $\sup\left\{\left(\partial f_{r}/\partial x_{r}\right)+\left(\partial f_{s}/\partial x_{s}\right)+\underset{q\neq r,s}{\Sigma }\left(\left|\partial f_{q}/\partial x_{r}\right|+\left|\partial f_{q}/\partial x_{s}\right|\right)\text{: }1\leq r<s\leq n\right\}<0$
- $\sup\left\{\left(\partial f_{r}/\partial x_{r}\right)+\left(\partial f_{s}/\partial x_{s}\right)+\underset{q\neq r,s}{\Sigma }\left(\left|\partial f_{r}/\partial x_{q}\right|+\left|\partial f_{s}/\partial x_{q}\right|\right)\text{: }1\leq r<s\leq n\right\}<0$
- *λ*_1_ + *λ*_2_ < 0
- $\inf\left\{\left(\partial f_{r}/\partial x_{r}\right)+\left(\partial f_{s}/\partial x_{s}\right)-\underset{q\neq r,s}{\Sigma }\left(\left|\partial f_{q}/\partial x_{r}\right|+\left|\partial f_{q}/\partial x_{s}\right|\right)\text{: }1\leq r<s\leq n\right\}>0$
- $\inf\left\{\left(\partial f_{r}/\partial x_{r}\right)+\left(\partial f_{s}/\partial x_{s}\right)-\underset{q\neq r,s}{\Sigma }\left(\left|\partial f_{r}/\partial x_{q}\right|+\left|\partial f_{s}/\partial x_{q}\right|\right)\text{: }1\leq r<s\leq n\right\}>0$
- *λ*_*n*−1_ + *λ*_*n*_ > 0

where *λ*_1_ ≥ *λ*_2_ ≥ *λ*_3_≥...≥*λ*_*n*_ are the eigenvalues of (1/2)((*∂f*/*∂x*)^∗^ + (*∂f*/*∂x*)) where ∗ denotes the transposition, and *∂f*/*∂x* is the Jacobian matrix of *f*.

The corresponding logarithmic norm of *J*^[2]^ is denoted by *μ*_∞_(*J*^[2]^) and provided by the vector norm |*x*| = sup_*i*_|*x*_*i*_| as follows:

(17) $$\begin{array}{c} \mu_{\infty }\left(J^{\left[2\right]}\right)=\sup\left\{\frac{\partial f_{r}}{\partial x_{r}}+\frac{\partial f_{s}}{\partial x_{s}}+\underset{q\neq r,s}{\Sigma }\left(\left|\frac{\partial f_{q}}{\partial x_{r}}\right|+\left|\frac{\partial f_{q}}{\partial x_{s}}\right|\right)\text{: }1\leq r<s\leq n\right\}, \end{array}$$

where *μ*_∞_(*J*^[2]^) < 0 implies the diagonal dominance by row matrix *J*^[2]^. Then, the following result holds.

**Theorem 9 .**

A simple closed rectifiable curve that is invariant under system (3) cannot exist [22] if *μ*_∞_(*J*^[2]^) < 0.

The nonexistence of periodic solutions of system (3) will be discussed by applying Li–Muldowney's criterion. The logarithm norm *μ*_∞_ of the second additive compound matrix *J*^[2]^, for the Jacobian *J*, is negative if the following conditions satisfy:

(18) $$\begin{array}{c} \frac{2\alpha S}{{\left(1+\delta I_{u}\right)}^{2}}-\left(\beta +\gamma +d_{1}+d_{2}\right)<0, \end{array}$$

(19) $$\begin{array}{c} \frac{\alpha }{{\left(1+\delta I_{u}\right)}^{2}}\left(S-I_{u}-\delta I_{u}^{2}\right)-2d_{1}<0, \end{array}$$

(20) $$\begin{array}{c} -\left(\gamma +d_{1}+d_{2}\right)<0, \end{array}$$

Now the left hand side of inequality (18)

(21) $$\begin{array}{c} \frac{2\alpha S}{{\left(1+\delta I_{u}\right)}^{2}}-\left(\beta +\gamma +d_{1}+d_{2}\right)\leq \beta +d_{1}-\gamma -d_{2}. \end{array}$$

Thus, inequality (18) will follow if *β* + *d*_1_ − *γ* − *d*_2_ < 0. So the inequalities (18), (19), and (20) can be easily demonstrated if (i), (ii), and (iii) hold, respectively, where (i)*β* + *d*_1_ − *γ* − *d*_2_ < 0, (ii)*d*_1_ > *β*, and (iii) *γ* + *d*_1_ + *d*_2_ > 0.

## 5. COVID-19 Model with Control

In this section, we extend the basic model (1) by including a particular control measure aimed at controlling the spread of the COVID-19 infection and formulate the optimal control problem by proposing the control objectives. The aim of the control measures is to reduce the infection in the population, and thus, there is the need to formulate the optimal control problem to achieve this goal. The control function *σ*(*t*) is applied as a vaccine for the susceptible, which reduces the number of infected people which spread the disease per unit of time. Under these control measure, the proposed model (1) is modified as

(22) $$\begin{array}{c} \begin{array}{c} \frac{dS}{dt}=\Lambda -\frac{\alpha S\left(t\right)I_{u}\left(t\right)}{1+\delta I_{u}\left(t\right)}-\sigma \left(t\right)S\left(t\right)-d_{1}S\left(t\right),\\ \frac{dI_{u}}{dt}=\frac{\alpha S\left(t\right)I_{u}\left(t\right)}{1+\delta I_{u}\left(t\right)}-\beta I_{u}\left(t\right)-d_{1}I_{u}\left(t\right),\\ \frac{dI_{k}}{dt}=\beta I_{u}\left(t\right)-\gamma I_{k}\left(t\right)-d_{2}I_{k}\left(t\right),\\ \frac{dR}{dt}=\sigma \left(t\right)S\left(t\right)+\gamma I_{k}\left(t\right)-d_{1}R\left(t\right), \end{array} \end{array}$$

with nonnegative initial conditions

(23) $$\begin{array}{c} S\left(0\right)={\overset{¯}{S}}_{0},R\left(0\right)={\overset{¯}{R}}_{0}>0,\\ I_{u}\left(0\right)={\overset{¯}{I}}_{u_{0}},I_{k}\left(0\right)={\overset{¯}{I}}_{k_{0}}\geq 0. \end{array}$$

The flow diagram of the proposed COVID-19 pandemic model with control is presented in Figure 3. The control is completely effective when *σ*(*t*) = 1, and the control is not effective when *σ*(*t*) = 0, i.e., 0 ≤ *σ*(*t*) ≤ 1. Our focus is to minimize the number of exposed individuals under the cost of applying control measures, which can be done by considering the following fractional optimal control problem to minimize the objective functional given by

(24) $$\begin{array}{c} J\left(\sigma \left(t\right)\right)=\int_{0}^{\tau }\left(Q_{1}S+\frac{1}{2}Q_{2}\sigma^{2}\right), \end{array}$$

subjected to the state system given in (22) along nonnegative initial conditions (23). In Equation (24), 𝒬_1_ and 𝒬_2_ represent the positive constants to keep a balance in the size of the terms. The square of the control variable reflects the severity of the side-effects of the vaccine. Our objective is to minimize the cost function *J*(*σ*(*t*)) given in (22) so that the spread of infection rate can be minimized. So, we seek an optimal control *σ*^∗^ such that

(25) $$\begin{array}{c} J\left(\sigma^{*}\right)=\min\left\{Y\left(\sigma \right)\text{: }\sigma \in U\right\}, \end{array}$$

subjected to the state system given in (22), where the control set is defined as

(26) $$\begin{array}{c} U=\left\{\left.\sigma \right|\sigma \left(t\right)\text{ is Lebesgue measurable on }\left[0,1\right]\right\}. \end{array}$$

### 5.1. Existence of an Optimal Control

**Lemma 1 .**

Every solution of system (22) with initial conditions (23) exists in the interval [0, ∞) and *S*(*t*) > 0, *I*_*u*_(*t*) ≥ 0, *I*_*k*_(*t*) ≥ 0, and *R*(*t*) > 0 for all *t* ≥ 0.

**Proof**

Since the right hand side of COVID-19 model (22) is continuous and locally Lipschitzian, then the solution (*S*(*t*), *I*_*u*_(*t*), *I*_*k*_(*t*), *R*(*t*)) of (22) using the initial conditions is unique on [0, *ξ*), where 0 < *ξ* < +∞.

From the model (22) and using the initial conditions, we have

(27) $$\begin{array}{c} \frac{dS}{dt}=\Lambda -\left(\sigma +d_{1}+\frac{\alpha I_{u}\left(t\right)}{1+\delta I_{u}\left(t\right)}\right)S\left(t\right). \end{array}$$

We thus have

(28) $$\begin{array}{c} \frac{d}{dt}\left[S\left(t\right)\exp\left\{\left(\sigma +d_{1}\right)t+\int_{0}^{t}\frac{\alpha I_{u}\left(s\right)}{1+\delta I_{u}\left(s\right)}ds\right\}\right]=\Lambda \exp\left\{\left(\sigma +d_{1}\right)t+\int_{0}^{t}\frac{\alpha I_{u}\left(s\right)}{1+\delta I_{u}\left(s\right)}ds\right\}. \end{array}$$

Hence,

(29) $$\begin{array}{c} S\left(t\right)\exp\left\{\left(\sigma +d_{1}\right)t+\int_{0}^{t}\frac{\alpha I_{u}\left(s\right)}{1+\delta I_{u}\left(s\right)}ds\right\}-S\left(0\right)=\int_{0}^{t}\Lambda \exp\left\{\left(\sigma +d_{1}\right)t+\int_{0}^{t}\frac{\alpha I_{u}\left(\omega \right)}{1+\delta I_{u}\left(\omega \right)}d\omega \right\}dt, \end{array}$$

so that

(30) $$\begin{array}{c} S\left(t\right)=S\left(0\right)\exp\left[-\left\{\left(\sigma +d_{1}\right)t+\int_{0}^{t}\frac{\alpha I_{u}\left(s\right)}{1+\delta I_{u}\left(s\right)}ds\right\}\right]+\exp\left[-\left\{\left(\sigma +d_{1}\right)t+\int_{0}^{t}\frac{\alpha I_{u}\left(s\right)}{1+\delta I_{u}\left(s\right)}ds\right\}\right]\times \left[\int_{0}^{t}\Lambda \exp\left\{\left(\sigma +d_{1}\right)t+\int_{0}^{t}\frac{\alpha I_{u}\left(\omega \right)}{1+\delta I_{u}\left(\omega \right)}d\omega \right\}dt\right]>0. \end{array}$$

The second equation of the model (22) yields

(31) $$\begin{array}{c} \frac{dI_{u}}{dt}\geq -\left(\beta +d_{1}\right)I_{u}\left(t\right), \end{array}$$

which provides *I*_*u*_(*t*) ≥ *I*_*u*_(0)exp[−(*β* + *d*_1_)*t*] ≥ 0.

From the third equation of system (1), we get

(32) $$\begin{array}{c} \frac{dI_{k}}{dt}\geq -\left(\gamma +d_{2}\right)I_{k}, \end{array}$$

which gives *I*_*k*_(*t*) ≥ *I*_*k*_(0)exp[−(*γ* + *d*_2_)*t*] ≥ 0.

Finally, the last equation of the system (22) yields

(33) $$\begin{array}{c} \frac{dR}{dt}\geq -d_{1}R\left(t\right), \end{array}$$

which provides *R*(*t*) ≥ *R*(0)exp[−(*d*_1_)*t*] > 0.

Therefore, we can see that *S*(*t*), *R*(*t*) > 0 and *I*_*u*_(*t*), *I*_*k*_(*t*) ≥ 0, ∀*t* ≥ 0. This completes the proof.

**Lemma 2 .**

All solutions of COVID-19 system (22) in ℝ_+_^4^ are bounded and lie in the region *Ω* defined by *Ω* = {(*S*, *I*_*u*_, *I*_*k*_, *R*) ∈ ℝ_+_^4^ : 0 < *N*(*t*) ≤ *Λ*/*μ*} as *t*⟶∞, where *μ* = min{*d*_1_, *d*_2_}.

**Proof**

Assume (*S*(*t*), *I*_*u*_(*t*), *I*_*k*_(*t*), *R*(*t*)) be any solution of system (22). Now, we consider a function like *N*(*t*) = *S*(*t*) + *I*_*u*_(*t*) + *I*_*k*_(*t*) + *R*(*t*). Differentiating both sides with respect to *t*, we have

(34) $$\begin{array}{c} \frac{dN\left(t\right)}{dt}=\frac{dS\left(t\right)}{dt}+\frac{dI_{u}\left(t\right)}{dt}+\frac{dI_{k}\left(t\right)}{dt}+\frac{dR\left(t\right)}{dt},\\ \frac{dN\left(t\right)}{dt}=\Lambda -d_{1}S-d_{1}I_{u}-d_{2}I_{k}-d_{1}R,\\ \frac{dN\left(t\right)}{dt}+\mu N\left(t\right)=\Lambda -\left(d_{1}-\mu \right)S-\left(d_{1}-\mu \right)I_{u}-\left(d_{2}-\mu \right)I_{k}-\left(d_{1}-\mu \right)R, \end{array}$$

(*dN*(*t*)/*dt*) + *μN*(*t*) ≤ *Λ*, assuming *μ* = min{*d*_1_, *d*_2_}.

Then by comparison theorem, we obtain 0 < *N*(*t*) ≤ *N*(0)*e*^−*μt*^ + (*Λ*/*μ*) and for *t*⟶∞, 0 < *N*(*t*) ≤ *Λ*/*μ*. Therefore, all solutions of coronavirus system (22) enter into the region *Ω* = {(*S*, *I*_*u*_, *I*_*k*_, *R*) ∈ ℝ_+_^4^ : 0 < *N*(*t*) ≤ *Λ*/*μ*}.

**Theorem 10 .**

Given the objective functional

(35) $$\begin{array}{c} J\left(\sigma \left(t\right)\right)=\int_{0}^{\tau }\left(Q_{1}S+\frac{1}{2}Q_{2}\sigma^{2}\right)dt, \end{array}$$

where *U* = {*σ*|*σ*(*t*) is Lebesgue measurable on [0, 1]} subject to the system [24] with [25], then there exists an optimal control *σ*^∗^ such that *J*(*σ*^∗^) = min{*Y*(*σ*): *σ* ∈ *U*}, if the following conditions are satisfied:

1. The class of all initial conditions with a control *σ*(*t*) in the admissible control set along with each state equation being satisfied is not empty
2. The admissible control set *U* is closed and convex
3. Each right hand side of the state system (22) is continuous and is bounded above by a sum of the bounded control and the state and can be written as a linear function of *σ* with coefficients depending on time and the state
4. The integrand of *J*(*σ*) is convex on *U* and is bounded below by *p*_1_*σ*^2^ − *p*_2_ with *p*_1_, *p*_2_ > 0

The proof is in the Appendix.

### 5.2. Characterization of the Optimal Control Pair

The Lagrangian *ℒ* and Hamiltonian *ℋ* for the fractional optimal problem Equations (22)–(26) are as follows:

(36) $$\begin{array}{c} L\left(S,\sigma \right)=Q_{1}S+\frac{Q_{2}}{2}\sigma^{2},\\ H\ll L\left(S,\sigma \right)+\lambda_{S}\frac{dS}{dt}+\lambda_{I_{u}}\frac{dI_{u}}{dt}+\lambda_{I_{k}}\frac{dI_{k}}{dt}+\lambda_{R}\frac{dR}{dt}. \end{array}$$

This further implies

(37) $$\begin{array}{c} H\ll Q_{1}S+\frac{Q_{2}}{2}\sigma^{2}+\lambda_{S}\left[\Lambda -\frac{\alpha S\left(t\right)I_{u}\left(t\right)}{1+\delta I_{u}\left(t\right)}-\sigma \left(t\right)S\left(t\right)-d_{1}S\left(t\right)\right]+\lambda_{I_{u}}\left[\frac{\alpha S\left(t\right)I_{u}\left(t\right)}{1+\delta I_{u}\left(t\right)}-\beta I_{u}\left(t\right)-d_{1}I_{u}\left(t\right)\right]+\lambda_{I_{k}}\left[\beta I_{u}\left(t\right)-\gamma I_{k}\left(t\right)-d_{2}I_{k}\left(t\right)\right]+\lambda_{R}\left[\sigma \left(t\right)S\left(t\right)+\gamma I_{k}\left(t\right)-d_{1}R\left(t\right)\right], \end{array}$$

where *λ*_*S*_, *λ*_*I*_*u*__, *λ*_*I*_*k*__, and *λ*_*R*_ are the adjoint variables to be determined suitably.

The forms of the adjoint equations and transversality conditions are standard results from Pontryagin's maximum principle. The adjoint system can be obtained as follows:

(38) $$\begin{array}{c} \begin{array}{cc} \lambda_{S}^{\prime } & =-\left(\frac{\partial H}{\partial S}\right)=\left(\lambda_{S}-\lambda_{I_{u}}\right)\frac{\alpha I_{u}}{1+\delta I_{u}}+d_{1}\lambda_{S}+\left(\lambda_{S}-\lambda_{R}\right)\sigma -Q_{1},\\ \lambda_{I_{u}}^{\prime } & =-\left(\frac{\partial H}{\partial I_{u}}\right)=\left(\lambda_{S}-\lambda_{I_{u}}\right)\frac{\alpha S}{{\left(1+\delta I_{u}\right)}^{2}}+\left(\beta +d_{1}\right)\lambda_{I_{u}}-\beta \lambda_{I_{k}},\\ \lambda_{I_{k}}^{\prime } & =-\left(\frac{\partial H}{\partial I_{k}}\right)=\left(\gamma +d_{2}\right)\lambda_{I_{k}}-\gamma \lambda_{R},\\ \lambda_{R}^{\prime } & =-\left(\frac{\partial H}{\partial R}\right)=d_{1}\lambda_{R}, \end{array} \end{array}$$

with transversality conditions or boundary conditions *λ*_*S*_(*τ*) = 0, *λ*_*I*_*u*__(*τ*) = 0, *λ*_*I*_*k*__(*τ*) = 0 and *λ*_*R*_(*τ*) = 0.

By the optimality condition, we have

(39) $$\begin{array}{c} \frac{\partial H}{\partial \sigma }=Q_{2}\sigma^{*}-\left(\lambda_{S}-\lambda_{R}\right){\overset{¯}{S}}^{*}=0\text{ at }\sigma =\sigma^{*}. \end{array}$$

By using the bounds for the control *σ*(*t*), we get

(40) $$\begin{array}{c} \sigma^{*}=\left\{\begin{array}{c} \frac{\left(\lambda_{S}-\lambda_{R}\right){\overset{¯}{S}}^{*}}{Q_{2}},\text{if }0\leq \frac{\left(\lambda_{S}-\lambda_{R}\right){\overset{¯}{S}}^{*}}{Q_{2}}\leq 1,\\ 0,\text{if}\frac{\left(\lambda_{S}-\lambda_{R}\right){\overset{¯}{S}}^{*}}{Q_{2}}\leq 0,\\ 1,\text{if}\frac{\left(\lambda_{S}-\lambda_{R}\right){\overset{¯}{S}}^{*}}{Q_{2}}\geq 1. \end{array}\right. \end{array}$$

In compact notation:

(41) $$\begin{array}{c} \sigma^{*}=\min\left\{\max\left(0,\frac{\left(\lambda_{S}-\lambda_{R}\right){\overset{¯}{S}}^{*}}{Q_{2}}\right),1\right\}. \end{array}$$

Using (22), we obtain the following optimality system:

(42) $$\begin{array}{c} \begin{array}{c} \frac{dS}{dt}=\Lambda -\frac{\alpha S\left(t\right)I_{u}\left(t\right)}{1+\delta I_{u}\left(t\right)}-\min\left\{\max\left(0,\frac{\left(\lambda_{S}-\lambda_{R}\right)S\left(t\right)}{Q_{2}}\right),1\right\}S\left(t\right)-d_{1}S\left(t\right),\\ \frac{dI_{u}}{dt}=\frac{\alpha S\left(t\right)I_{u}\left(t\right)}{1+\delta I_{u}\left(t\right)}-\beta I_{u}\left(t\right)-d_{1}I_{u}\left(t\right),\\ \frac{dI_{k}}{dt}=\beta I_{u}\left(t\right)-\gamma I_{k}\left(t\right)-d_{2}I_{k}\left(t\right),\\ \frac{dR}{dt}=\min\left\{\max\left(0,\frac{\left(\lambda_{S}-\lambda_{R}\right)S\left(t\right)}{Q_{2}}\right),1\right\}S\left(t\right)+\gamma I_{k}\left(t\right)-d_{1}R\left(t\right),\\ \frac{d\lambda_{S}}{dt}=\left(\lambda_{S}-\lambda_{I_{u}}\right)\frac{\alpha I_{u}}{1+\delta I_{u}}+d_{1}\lambda_{S}-Q_{1}+\left(\lambda_{S}-\lambda_{R}\right)\min\left\{\max\left(0,\frac{\left(\lambda_{S}-\lambda_{R}\right)S\left(t\right)}{Q_{2}}\right),1\right\},\\ \frac{d\lambda_{I_{u}}}{dt}=\left(\lambda_{S}-\lambda_{I_{u}}\right)\frac{\alpha S}{{\left(1+\delta I_{u}\right)}^{2}}+\left(\beta +d_{1}\right)\lambda_{I_{u}}-\beta \lambda_{I_{k}},\\ \frac{d\lambda_{I_{k}}}{dt}=\left(\gamma +d_{2}\right)\lambda_{I_{k}}-\gamma \lambda_{R},\\ \frac{d\lambda_{R}}{dt}=d_{1}\lambda_{R}, \end{array} \end{array}$$

with nonnegative initial conditions

(43) $$\begin{array}{c} S\left(0\right)>0,I_{u}\left(0\right)\geq 0,R\left(0\right)>0,I_{k}\left(0\right)\geq 0,\\ \lambda_{S}\left(\tau \right)=0,\lambda_{I_{u}}\left(\tau \right)=0,\lambda_{I_{k}}\left(\tau \right)=0,\lambda_{R}\left(\tau \right)=0. \end{array}$$

The previous analysis can be summarized in the following theorem.

**Theorem 11 .**

Let ${\overset{¯}{S}}^{*},{\overset{¯}{I}}_{u}^{*},{\overset{¯}{I}}_{k}^{*}$, and ${\overset{¯}{R}}^{*}$ be optimal state solutions with associated optimal control variable *σ*^∗^ for the optimal control problems (22) and (23). Then there exist adjoint variables *λ*_*S*_, *λ*_*I*_*u*__, *λ*_*I*_*k*__, and *λ*_*R*_ satisfying

(44) $$\begin{array}{c} \begin{array}{c} \lambda_{S}^{\prime }=-\left(\frac{\partial H}{\partial S}\right)=\left(\lambda_{S}-\lambda_{I_{u}}\right)\frac{\alpha I_{u}}{1+\delta I_{u}}+d_{1}\lambda_{S}+\left(\lambda_{S}-\lambda_{R}\right)\sigma -Q_{1},\\ \lambda_{I_{u}}^{\prime }=-\left(\frac{\partial H}{\partial I_{u}}\right)=\left(\lambda_{S}-\lambda_{I_{u}}\right)\frac{\alpha S}{{\left(1+\delta I_{u}\right)}^{2}}+\left(\beta +d_{1}\right)\lambda_{I_{u}}-\beta \lambda_{I_{k}},\\ \lambda_{I_{k}}^{\prime }=-\left(\frac{\partial H}{\partial I_{k}}\right)=\left(\gamma +d_{2}\right)\lambda_{I_{k}}-\gamma \lambda_{R},\\ \lambda_{R}^{\prime }=-\left(\frac{\partial H}{\partial R}\right)=d_{1}\lambda_{R}, \end{array} \end{array}$$

with transversality conditions or boundary conditions *λ*_*S*_(*τ*) = 0, *λ*_*I*_*u*__(*τ*) = 0, *λ*_*I*_*k*__(*τ*) = 0 and *λ*_*R*_(*τ*) = 0.

Furthermore, the control functions *σ*^∗^ is given by

(45) $$\begin{array}{c} \sigma^{*}=\min\left\{\max\left(0,\frac{\left(\lambda_{S}-\lambda_{R}\right){\overset{¯}{S}}^{*}}{Q_{2}}\right),1\right\}. \end{array}$$

**Proof**

The adjoint system (42), i.e., *λ*_*S*_′, *λ*_*I*_*u*__′, *λ*_*I*_*k*__′, and *λ*_*R*_′, is obtained from the Hamiltonian *ℋ* as

(46) $$\begin{array}{c} -\frac{d\lambda_{S}}{dt}=\frac{\partial H}{\partial S},-\frac{d\lambda_{I_{u}}}{dt}=\frac{\partial H}{\partial I_{u}},-\frac{d\lambda_{I_{k}}}{dt}=\frac{\partial H}{\partial I_{k}},-\frac{d\lambda_{R}}{dt}=\frac{\partial H}{\partial R}, \end{array}$$

with zero final time conditions (transversality), conditions *λ*_*S*_(*τ*) = 0, *λ*_*I*_*u*__(*τ*) = 0, *λ*_*I*_*k*__(*τ*) = 0 and *λ*_*R*_(*τ*) = 0, and the characterization of the fractional optimal control given by (45) is obtained by solving the equation *∂ℋ*/*∂σ* = 0 on the interior of the control set and using the property of the control space *U*.

Hence, that is the theorem.

## 6. Numerical Demonstration

The numerical part of this paper is introduced to obtain some sound results based on some data using MATLAB. For parameter estimation, we have not used any mathematical method; we use the trial and error method to fit our model to the actual data. This work intends not to find the exact value of the parameter; we want to see the hidden fact of the outspread speed. We consider a small amount for the initial condition of the susceptible population in both waves, and our model almost represents the same result as accurately (Figures 4–7). That is an exciting result that COVID is not homogeneously spread all over India and we can control it by lockdown. However, lockdown can pull down the economy, which is an extensive issue to use this method. Our study hints that another technique to control is to find unrevealed COVID patients as early as possible (Figures 8 and 9). The detected patients are not major responsible for the spread, rather the unrevealed patient mainly spreads COVID. Another question that has a great impact on society is that how many waves face India? The answer depends on the vaccination speed and the variant; however, mathematically, we did not find multiple waves from a single COVID-19 variant. If vaccines work for all variants, then this is the first and last strategy to defend COVID-19 and various waves. If we do not complete the vaccination within the ongoing wave, then we may face the next wave, and so on. Moreover, the community of poor, uneducated, insanitary, and highly dense populations would not control waves without vaccine help. Another question that can answer our model is what will be the peak value of the subsequent consequence wave? The answer is straightforward; the peak value always crosses its past value because COVID spreads from big town to small town to the village in successive waves (see Figures 10 and 11). We draw the figures from Figures 4–13 based on the parameter value and initial condition for both waves using Tables 1 and 2. For Figure 5, we take *I*_*u*_(0) = 70000 and the rest of the initial values and parameter values are the same shown in Tables 1 and 2. For our study, we take statistical data from https://www.worldometers.info/ [26].

Our chosen parameter set of the model by trial and error method almost satisfies the actual situation.  Figure 4 represents the known and unrevealed infected population in the first wave and Figure 5 for the second wave.  Figure 6 is for the susceptible and recover class for the 1st wave and Figure 7 is for the 2nd wave. The 1st and 2nd wave end their journey. We studied them to know the hidden dynamics. Our numerical study satisfies our model assuming the unknown infected population is critical for spreading the disease. So controlling the 3rd wave is a big challenge for India due to its vast population.

Figure 8 for the 1st wave and Figure 9 for the 2nd wave show exciting findings. If we can identify unknown infected people quickly, then we can control COVID spread effectively; however, it is a difficult job for a country with a large population. Figures 10 and 11 for the 1st and 2nd wave, respectively, answer the effectiveness of lockdown. Implementing lockdown can only control the spread more effectively since the initial population for the susceptible variable will be small. Figures 12 and 13 for the 1st and 2nd wave, respectively, show the psychological effect on COVID propagation. Media-created fear on the human population has a clear impact on propagation.

### 6.1. Optimal Control

Here, we use some numerical simulations to investigate the effect of the suggested control strategy, vaccine, on the outbreak of COVID-19. From Figure 14, it is clear that when time increases, then optimal vaccine control strategies decreases time to time in a country like India. It is clear that the vaccine reduces the number of infected people. Figure 14 shows the speed of vaccination to control the disease within 30 days. This is mathematical analysis; reality is complicated. To prevent illness within 30 days, massive vaccine and huge trained human experts are required. Figures 15 plots the variation in the number of susceptible, unrevealed infected, known infected, and recovery people in the presence and the absence of the control strategy in India. Our goal was to reduce the number of infected people; the results confirm that the number of infected people decreased, and since the initial number of infected people was small, this wave ended faster, and the spread of the disease was controlled by the vaccine strategy. We use Tables 2 and 3 (2nd wave) to present Figures 14 and 15 for the model with controls (22).

## 7. Observations and Conclusion

This paper has proposed a model for infectious novel coronavirus disease for the dynamical study. The BRN *R*_0_ is the threshold condition that determines the disease propagation dynamics. This study has shown that when *R*_0_ < 1, the system has only a globally stable disease-free equilibrium *E*_1_ which leads to the eventual death of the disease. The coronavirus system has a unique endemic equilibrium *E*^∗^ for *R*_0_ > 1, which is globally stable under the same condition. In this paper, mainly we consider data of two different waves in India and checked which of the waves is more dangerous in India. We checked the effect of different parameters through the figures; the truth tells that the second wave is more dangerous than the first wave. The next focus of this paper is to set up an optimal control problem relative to the COVID-19 epidemic model to minimize the daily infected people. We have considered the vaccine rate as a function of time by *σ*(*t*). *σ* is representing the vaccine control in this COVID model. The control function *σ* is designed in such a way that it minimizes the objective functional (cost function) *J* as given in [27]. Finally, we found some exciting results by studying the presented model numerically based on accurate data. Lockdown is the best technique mathematically to control the disease spread. However, ideal lockdown is not possible in practice, so we did not find satisfying practical results by using this method. These measures have proven unpopular due to their social and economic consequences, so it is essential to find new standards. Quick detection of undetected patents can control the spread. Vaccination can handle the situation; otherwise, we observe many waves. Mathematically, we did not find multiple waves from a single COVID-19 variant since the new variants produce distinct waves. If vaccines work for each variant, this is the most acceptable strategy to defend the various upcoming waves. We have monitored the psychological effect on infection propagation. This study has observed that media-created fear negatively affects human psychology and affects COVID dynamics positively. The peak value of subsequent consequence waves always crosses its past value because this disease spreads from the big town to the small town to the village in successive waves, and new strains are more quickly spread than the previous version.

## Figures and Tables

**Figure 1:** Transfer diagram of the proposed COVID-19 system.

**Figure 2:** Change of *ℜ*_0_ with respect to *α* in two different waves using data in Table 1.

**Figure 3:** Transfer diagram of COVID-19 model with control.

**Figure 4:** Time graph of the first wave of unrevealed infected population (*I*_*u*_) and known infected population (*I*_*k*_) for *α* = 54 × 10^−10^, *α* = 55 × 10^−10^, and *α* = 56 × 10^−10^ in India.

**Figure 5:** Second wave time graph of unrevealed infected population (*I*_*u*_) and known infected population (*I*_*k*_) for *α* = 54 × 10^−10^, *α* = 55 × 10^−10^, and *α* = 56 × 10^−10^ in India.

**Figure 6:** Time history of the susceptible (*S*) and recovery population (*R*) of the first wave for *α* = 54 × 10^−10^, *α* = 55 × 10^−10^, and *α* = 56 × 10^−10^ in India.

**Figure 7:** Time graph of the second wave for susceptible (*S*) and recovery population (*R*) for *α* = 54 × 10^−10^, *α* = 55 × 10^−10^, and *α* = 56 × 10^−10^ in India.

**Figure 8:** Time history of unrevealed infected population (*I*_*u*_) and known infected population (*I*_*k*_) of the first wave for *β* = 0.20, *β* = 0.21, and *β* = 0.22 in India.

**Figure 9:** Time history of unrevealed infected population (*I*_*u*_) and known infected population of the second wave (*I*_*k*_) for *β* = 0.20, *β* = 0.21, and *β* = 0.22 in India.

**Figure 10:** First wave time history of unrevealed infected population (*I*_*u*_) and known infected population (*I*_*k*_) for *S*_0_ = 5 × 10^7^, *S*_0_ = 6 × 10^7^, and *S*_0_ = 7 × 10^7^ in India.

**Figure 11:** Time history of unrevealed infected population (*I*_*u*_) and known infected population of the second wave (*I*_*k*_) for *S*_0_ = 6 × 10^7^, *S*_0_ = 7 × 10^7^, and *S*_0_ = 8 × 10^7^ in India.

**Figure 12:** First wave time history of unrevealed infected population (*I*_*u*_) and known infected population (*I*_*k*_) for *δ* = 25 × 10^−8^, *δ* = 33 × 10^−8^, and *δ* = 4 × 10^−7^ in India.

**Figure 13:** Time history of unrevealed infected population (*I*_*u*_) and known infected population of the second wave (*I*_*k*_) for *δ* = 1 × 10^−7^, *δ* = 135 × 10^−9^, and *δ* = 17 × 10^−8^ in India.

**Figure 14:** The optimal control diagrams for the vaccine control, with input values from Table 3.

**Figure 15:** Plots for *S*, *I*_*u*_, *I*_*k*_, and *R* in the presence and absence of control using data from Table 3.

**Table 1:** Explanation of parameters with their real field value.

Parameters	Interpretation	Value of the 1st wave/day	Value of the 2nd wave/day	Reference
*Λ*	Recruitment rate of new individuals	1 × 10^3^	2 × 10^3^	Fitted
*α*	Transmission coefficient from SP to *I*_*u*_P	55 × 10^−10^	55 × 10^−10^	Fitted
*δ*	Measures of the psychological or inhibitory effect	33 × 10^−8^	135 × 10^−9^	Fitted
*β*	Transmission coefficient from *I*_*u*_P to *I*_*k*_P	0.21	0.21	Fitted
*γ*	Transmission coefficient from *I*_*k*_P to RP	0.1	0.1	Fitted
*d*_1_	Natural death rate	4 × 10^−5^	4 × 10^−5^	Fitted
*d*_2_	Death rate due to COVID-19 plus *d*_1_	1 × 10^−3^	1 × 10^−3^	Fitted

**Table 2:** Initial population for different waves.

Initial population	Initial value for the 1st wave	Initial value for the 2nd wave
*S*(0)	5 × 10^7^	6 × 10^7^
*I*_*u*_(0)	250	15 × 10^4^
*I*_*k*_(0)	256	170126

**Table 3:** Parameter values for the optimal control problem.

Parameters	Value per day
*Λ*	2 × 10^3^
*α*	55 × 10^−10^
*δ*	135 × 10^−9^
*β*	0.21
*γ*	0.1
*d*_1_	4 × 10^−5^
*d*_2_	1 × 10^−3^
𝒬_1_	40
𝒬_2_	1 × 10^5^

## Data Availability

The data used to support the findings of this study are available from the corresponding author upon request.

## Appendix

### A. Proof of Theorem 4

Proof The variational matrix of COVID-19 system (3) at *E*_1_(*Λ*/*d*_1_, 0, 0) is given by

(A.1) $$\begin{array}{c} V\left(E_{1}\right)=\left(\begin{array}{ccc} -d_{1} & -\frac{\alpha \Lambda }{d_{1}} & 0\\ 0 & \frac{\alpha \Lambda }{d_{1}}-\left(\beta +d_{1}\right) & 0\\ 0 & \beta & -\left(\gamma +d_{2}\right) \end{array}\right). \end{array}$$

The eigenvalues of the characteristic equation of *V*(*E*_1_) are obtained as *λ*_1_ = −*d*_1_ < 0, *λ*_2_ = (*αΛ*/*d*_1_) − (*β* + *d*_1_), and *λ*_3_ = −(*γ* + *d*_2_) < 0. Therefore, disease-free equilibrium point *E*_1_(*Λ*/*d*_1_, 0, 0) is locally asymptotically stable if *λ*_2_ = (*αΛ*/*d*_1_) − (*β* + *d*_1_) < 0, i.e., *ℜ*_0_ = *αΛ*/((*β* + *d*_1_)*d*_1_) < 1. Equilibrium point is marginally stable if *λ*_2_ = (*αΛ*/*d*_1_) − (*β* + *d*_1_) = 0, i.e., *R*_0_ = *αΛ*/(*β* + *d*_1_)*d*_1_ = 1. Equilibrium point is unstable if *λ*_2_ = (*αΛ*/*d*_1_) − (*β* + *d*_1_) > 0, i.e., *ℜ*_0_ = *αΛ*/(*β* + *d*_1_)*d*_1_ > 1. This completes the proof.

### B. Proof of Theorem 5

Proof The variational matrix of system (3) at *E*^∗^(*S*^∗^, *I*_*u*_^∗^, *I*_*k*_^∗^) is given by

(B.1) $$\begin{array}{c} V\left(E^{*}\right)=\left(\begin{array}{ccc} p_{11} & p_{12} & p_{13}\\ p_{21} & p_{22} & p_{23}\\ p_{31} & p_{32} & p_{33} \end{array}\right), \end{array}$$

where *p*_11_ = −(*αI*_*u*_^∗^/(1 + *δI*_*u*_^∗^)) − *d*_1_, *p*_12_ = −*αS*^∗^/(1 + *δI*_*u*_^∗^)^2^, *p*_13_ = 0, *p*_21_ = *αI*_*u*_^∗^/(1 + *δI*_*u*_^∗^), *p*_22_ = (*αS*^∗^/(1 + *δI*_*u*_^∗^)^2^) − (*β* + *d*_1_), *p*_23_ = 0, *p*_31_ = 0, *p*_32_ = *β*, *p*_33_ = −(*γ* + *d*_2_). Therefore, the characteristic equation of *V*(*E*^∗^) is

(B.2) $$\begin{array}{c} \left(\lambda -p_{33}\right)\left(\lambda^{2}+m_{1}\lambda +m_{2}\right)=0, \end{array}$$

where *p*_33_ = −(*γ* + *d*_2_) < 0, *m*_1_ = −(*p*_11_ + *p*_22_) = ((*α* + *δ*(*β* + *d*_1_))*I*_*u*_^∗^/(1 + *δI*_*u*_^∗^)) + *d*_1_ > 0, *m*_2_ = (*p*_11_*p*_22_ − *p*_12_*p*_21_) = [*αΛ* − *d*_1_(*β* + *d*_1_)]((*α* + *δ*)(*β* + *d*_1_)/*α*(*δΛ* + *β* + *d*_1_)). Based on Routh–Hurwitz criterion, the eigenvalues of Equation (B2) have negative real parts if [*αΛ* − *d*_1_(*β* + *d*_1_)] > 0, i.e., *ℜ*_0_ = *αΛ*/(*β* + *d*_1_)*d*_1_ > 1. Therefore, the endemic equilibrium point *E*^∗^ is locally asymptotically stable when *ℜ*_0_ > 1.

### C. Proof of Theorem 6

Proof The system (3) can be rewritten as

(C.1) $$\begin{array}{c} \begin{array}{c} \frac{dX}{dt}=F\left(X,Y\right),\\ \frac{dY}{dt}=G\left(X,Y\right),G\left(X,0\right)=0, \end{array} \end{array}$$

where *X* = *S* ∈ *R* stands for the number of uninfected individuals and *Y* = (*I*_*u*_, *I*_*k*_) ∈ *R*^2^ denotes the number of infected individuals. *U*_0_ = (*X*^∗^, 0) = *E*_1_(*Λ*/*d*_1_, 0, 0) shows the disease-free equilibrium of COVID-19 system. The global stability of the disease-free equilibrium *E*_1_ will guarantee upon the satisfaction of the following two conditions:

1. For *dX*/*dt* = *F*(*X*, 0), *X*^∗^ is globally asymptotically stable
2. $G\left(X,Y\right)=AY-\tilde{G}\left(X,Y\right),$$\tilde{G}\left(X,Y\right)\geq 0$, for (*X*, *Y*) ∈ *Ω*

where *A* = *D*_*Y*_*G*(*X*^∗^, 0) is Metzler matrix and *Ω* is the region of biological sense of the model. Following Castillo-Chavez et al. [28], we check for the aforementioned conditions. For the system (3), *F*(*X*, 0) = *Λ* − (*d*_1_)*S*,

(C.2) $$\begin{array}{c} A=\left(\begin{array}{cc} \frac{\Lambda \alpha }{d_{1}}-\left(\beta +d_{1}\right) & 0\\ \beta & -\left(\gamma +d_{2}\right) \end{array}\right),\\ \tilde{G}\left(X,Y\right)=\left(\begin{array}{c} \frac{\alpha \delta SI_{u}^{2}}{1+\delta I_{u}}\\ 0 \end{array}\right)\geq 0. \end{array}$$

As the off diagonal elements of *A* are nonnegative and $\tilde{G}\left(X,Y\right)\geq 0$, hence the disease-free equilibrium *E*_1_ is globally asymptotically stable if *ℜ*_0_ < 1.

### D. Proof of Theorem 8

Proof Since *S*(*t*) + *I*_*u*_(*t*) + *I*_*k*_(*t*) + *R*(*t*) = *N*(*t*), then it is adequate for the dynamical study of the three-dimensional COVID-19 system following:

(D.1) $$\begin{array}{c} \begin{array}{c} \frac{dS}{dt}=\Lambda -\frac{\alpha SI_{u}}{1+\delta I_{u}}-d_{1}S,\\ \frac{dI_{u}}{dt}=\frac{\alpha SI_{u}}{1+\delta I_{u}}-\beta I_{u}-d_{1}I_{u},\\ \frac{dI_{k}}{dt}=\beta I_{u}-\gamma I_{k}-d_{2}I_{k}. \end{array} \end{array}$$

The Jacobian matrix of the system (D1) is

(D.2) $$\begin{array}{c} J=\left(\begin{array}{ccc} p_{11} & p_{12} & p_{13}\\ p_{21} & p_{22} & p_{23}\\ p_{31} & p_{32} & p_{33} \end{array}\right)=\left(\begin{array}{ccc} -\frac{\alpha I_{u}}{1+\delta I_{u}}-d_{1} & -\frac{\alpha S}{{\left(1+\delta I_{u}\right)}^{2}} & 0\\ \frac{\alpha I_{u}}{1+\delta I_{u}} & \frac{\alpha S}{{\left(1+\delta I_{u}\right)}^{2}}-\left(\beta +d_{1}\right) & 0\\ 0 & \beta & -\left(\gamma +d_{2}\right) \end{array}\right). \end{array}$$

The associated second compound matrix is given by

(D.3) $$\begin{array}{c} J^{\left[2\right]}=\left(\begin{array}{ccc} p_{11}+p_{22} & p_{23} & -p_{13}\\ p_{32} & p_{11}+p_{33} & p_{12}\\ -p_{31} & p_{21} & p_{22}+p_{33} \end{array}\right), \end{array}$$

where *p*_11_ + *p*_22_ = −(*αI*_*u*_/1 + *δI*_*u*_) + (*αS*/(1 + *δI*_*u*_)^2^) − (*d*_1_ + *β* + *d*_1_), *p*_23_ = *p*_13_ = *p*_31_ = 0, *p*_32_ = *β*, *p*_11_ + *p*_33_ = −(*αI*_*u*_/1 + *δI*_*u*_) − (*d*_1_ + *γ*_2_ + *d*_2_), *p*_12_ = −*αS*/(1 + *δI*_*u*_)^2^, *p*_21_ = *αI*_*u*_/1 + *δI*_*u*_, *p*_22_ + *p*_33_ = (*αS*/(1 + *δI*_*u*_)^2^) − (*β* + *γ* + *d*_1_ + *d*_2_). We set the matrix function *A* by *A* = diag{1, *I*_*u*_/*I*_*k*_, *I*_*u*_/*I*_*k*_}. Then, *A*_*f*_*A*^−1^ = diag{0, (*I*_*u*_′/*I*_*u*_) − (*I*_*k*_′/*I*_*k*_), (*I*_*u*_′/*I*_*u*_) − (*I*_*k*_′/*I*_*k*_)}. We obtain the matrix *Q* in the block form as

(D.4) $$\begin{array}{c} Q_{3\times 3}=A_{f}A^{-1}+AJ^{\left[2\right]}A^{-1}=\left(\begin{array}{cc} Q_{11} & Q_{12}\\ Q_{21} & Q_{22} \end{array}\right), \end{array}$$

where $Q_{11}=-\left(\alpha I_{u}/1+\delta I_{u}\right)+\left(\alpha S/{\left(1+\delta I_{u}\right)}^{2}\right)-\left(2d_{1}+\beta \right),Q_{12}=\left(0\;0\right),Q_{21}=\left(\begin{array}{c} \left(I_{u}/I_{k}\right)\beta \\ 0 \end{array}\right)$,

(D.5) $$\begin{array}{c} Q_{22}=\left(\begin{array}{cc} \frac{I_{u}^{\prime }}{I_{u}}-\frac{I_{k}^{\prime }}{I_{k}}-\frac{\alpha I_{u}}{1+\delta I_{u}}-\left(2d_{1}+\gamma \right) & -\frac{\alpha S}{{\left(1+\delta I_{u}\right)}^{2}}\\ \frac{\alpha I_{u}}{1+\delta I_{u}} & \frac{I_{u}^{\prime }}{I_{u}}-\frac{I_{k}^{\prime }}{I_{k}}+\frac{\alpha S}{{\left(1+\delta I_{u}\right)}^{2}}-\left(\beta +\gamma +d_{1}+d_{2}\right) \end{array}\right). \end{array}$$

The vector norm |.| in ℝ^3^ can be chosen as |(*u*, *v*, *w*)| = max{|*u*|, |*v*| + |*w*|}. Let *μ* denote the Lozinskii measure [22] with respect to this norm. Then, we can obtain *μ*(*Q*) ≤ sup{*g*_1_, *g*_2_}, with *g*_1_ = *μ*_1_(*Q*_11_) + |*Q*_12_|, *g*_2_ = *μ*_1_(*Q*_22_) + |*Q*_21_|, where |*Q*_12_|, |*Q*_21_| are matrix norms with respect to the *L*^1^ vector norm and *μ*_1_ denotes the Lozenskii measure with respect to the *L*^1^ norm. Specifically, *μ*_1_(*Q*_11_) = (*αS*/(1 + *δI*_*u*_)^2^) − (*αI*_*u*_/1 + *δI*_*u*_) − (2*d*_1_ + *β*), |*Q*_12_| = max{0, 0} = 0, |*Q*_21_| = (*I*_*u*_/*I*_*k*_)*β*,

(D.6) $$\begin{array}{c} \mu_{1}\left(Q_{22}\right)=\frac{I_{u}^{\prime }}{I_{u}}-\frac{I^{\prime }}{I_{k}}-\gamma_{2}-d_{2}+\max\left\{-d_{1},\frac{2\alpha S}{{\left(1+\delta I_{u}\right)}^{2}}-\beta -d_{1}\right\}. \end{array}$$

Since (*αS*/(1 + *δI*_*u*_)^2^) − (*β* + *d*_1_) + |−*αS*/(1 + *δI*_*u*_)^2^| ≤ −*d*_1_, therefore *μ*_1_(*Q*_22_) = (*I*_*u*_′/*I*_*u*_) − (*I*′/*I*_*k*_) − *γ* − *d*_1_ − *d*_2_, and we have *g*_1_ = (*αS*/(1 + *δI*_*u*_)^2^) − (*αI*_*u*_/1 + *δI*_*u*_) − (2*d*_1_ + *β*). It follows from (12) that *I*_*u*_′/*I*_*u*_ = (*αS*/(1 + *δI*_*u*_)) − (*β* + *d*_1_). It implies *g*_1_ = (*I*_*u*_′/*I*_*u*_) − *d*_1_ − (*αI*_*u*_/1 + *δI*_*u*_) + (*αS*/(1 + *δI*_*u*_)^2^) − (*αS*/(1 + *δI*_*u*_)) ≤ (*I*_*u*_′/*I*_*u*_) − *d*_1_, *g*_2_ = (*I*_*u*_′/*I*_*u*_) − (*I*_*k*_′/*I*_*k*_) − *γ* − *d*_2_ + (*I*_*u*_*β*/*I*_*k*_) + max{−*d*_1_, (2*αS*/(1 + *δI*_*u*_)^2^) − *β* − *d*_1_}. Based on Equation (12), we have *I*_*k*_′/*I*_*k*_ = (*I*_*u*_*β*/*I*_*k*_) − *γ* − *d*_2_; hence, we get *g*_2_ ≤ (*I*_*u*_′/*I*_*u*_) − *d*_1_. Therefore, *μ*(*Q*) ≤ (*I*_*u*_′/*I*_*u*_) − *d*_1_. Thus, for *t* > *T*, we have (1/*t*)∫_0_^*t*^*μ*(*Q*)*ds* ≤ (1/*t*)log(*I*_*u*_′(*t*)/*I*_*u*_(*t*)) + (1/*t*)∫_0_^*T*^*μ*(*Q*)*ds* − ((*t* − *T*)*d*_1_/*t*), which implies ${\overset{¯}{q}}_{2}<0$. This completes the proof.

### E. Proof of Theorem 13

Proof In order to verify the first condition, we use a result by Lukes [29] (Theorem 9.2.1) for the system (22) with bounded coefficients. The control set *U* is convex and closed by definition, which gives condition (2). Therefore, the right hand side of the state system (22) satisfies condition (3) as the state solutions are prior bounded (see Lemmas 11 and 12). For the fourth condition, we need to show

(E.1) $$\begin{array}{c} g\left(\left(1-p\right)u+pv\right)\leq \left(1-p\right)g\left(u\right)+pg\left(v\right), \end{array}$$

where *g*(*x*) = 𝒬_1_*S* + (1/2)𝒬_2_*x*^2^. Now,

(E.2) $$\begin{array}{c} g\left(\left(1-p\right)u+pv\right)-\left[\left(1-p\right)g\left(u\right)+pg\left(v\right)\right]=Q_{1}S\left(t\right)+\frac{Q_{2}}{2}{\left\{\left(1-p\right)u+pv\right\}}^{2}-\left[\left(1-p\right)\left\{Q_{1}S\left(t\right)+\frac{Q_{2}}{2}u^{2}\right\}+p\left\{Q_{1}S\left(t\right)+\frac{Q_{2}}{2}v^{2}\right\}\right]=\frac{Q_{2}}{2}\left(p^{2}-p\right){\left(u-v\right)}^{2}. \end{array}$$

Since *p* ∈ (0, 1) implies (*p*^2^ − *p*) ≤ 0 and (*u* − *v*)^2^ > 0, the expression (𝒬_2_/2)(*p*^2^ − *p*)(*u* − *v*)^2^ ≤ 0, which implies that *g*((1 − *p*)*u* + *pv*) ≤ (1 − *p*)*g*(*u*) + *pg*(*v*). Lastly, 𝒬_1_*S*(*t*) + (𝒬_2_/2)*σ*^2^ ≥ (𝒬_2_/2)*σ*^2^(*t*) ≥ (𝒬_2_/2)*σ*^2^(*t*) − *p*_2_ ≥ *p*_1_*σ*^2^(*t*) − *p*_2_, which gives *p*_1_*σ*^2^(*t*) − *p*_2_ as a lower bound of *g*(*u*), for some *p*_1_ > 0, *p*_2_ > 0. Therefore, we can conclude that there exists an optimal control *σ*^∗^ such that *J*(*σ*^∗^) = min{*Y*(*σ*): *σ* ∈ *U*}.
